This article has been retracted.

# Heteroatoms (Si, B, N, and P) doped 2D monolayer MoS_2_ for NH_3_ gas detection†

**DOI:** 10.1039/d2ra04028j

**Published:** 2022-09-13

**Authors:** Terkumbur E. Gber, Hitler Louis, Aniekan E. Owen, Benjamin E. Etinwa, Innocent Benjamin, Fredrick C. Asogwa, Muyiwa M. Orosun, Ededet A. Eno

**Affiliations:** Computational and Bio-Simulation Research Group, University of Calabar Calabar Nigeria louismuzong@gmail.com; Department of Pure and Applied Chemistry, Faculty of Physical Sciences, University of Calabar Calabar Nigeria; Department of Chemistry, Akwa-Ibom State University Uyo Nigeria; Department of Physics, University of Ilorin Ilorin Nigeria

## Abstract

2D transition metal dichalcogenide MoS_2_ monolayer quantum dots (MoS_2_-QD) and their doped boron (B@MoS_2_-QD), nitrogen (N@MoS_2_-QD), phosphorus (P@MoS_2_-QD), and silicon (Si@MoS_2_-QD) surfaces have been theoretically investigated using density functional theory (DFT) computation to understand their mechanistic sensing ability, such as conductivity, selectivity, and sensitivity toward NH_3_ gas. The results from electronic properties showed that P@MoS_2_-QD had the lowest energy gap, which indicated an increase in electrical conductivity and better adsorption behavior. By carrying out comparative adsorption studies using m062-X, ωB97XD, B3LYP, and PBE0 methods at the 6-311G++(d,p) level of theory, the most negative values were observed from ωB97XD for the P@MoS_2_-QD surface, signifying the preferred chemisorption surface for NH_3_ detection. The mechanistic studies provided in this study also indicate that the P@MoS_2_-QD dopant is a promising sensing material for monitoring ammonia gas in the real world. We hope this research work will provide informative knowledge for experimental researchers to realize the potential of MoS_2_ dopants, specifically the P@MoS_2_-QD surface, as a promising candidate for sensors to detect gas.

## Abstract 2

2D transition metal dichalcogenide MoS_2_ monolayer quantum dots (MoS_2_-QD) and their doped boron (B@MoS_2_-QD), nitrogen (N@MoS_2_-QD), phosphorus (P@MoS_2_-QD), and silicon (Si@MoS_2_-QD) counterparts are proposed as selective sensors for NH_3_ gas.

## 1. Introduction

Molybdenum disulfide (MoS_2_) a 2D transition metal dichalcogenide (TMD), has attracted great scientific interest due to its intrinsic band gap compared to 2D materials like graphene which has a zero band gap.^1,2^ Due to the intrinsic band gap of MoS_2_ and its optoelectronic properties, it has been found to have interesting characteristics, such as high sensitivity, fast response, high selectivity, good reliability, quick recovery, high specific surface area, good chemical stability, high thermal stability and high surface activity compared to other 2D materials. These features and many more have drawn the attention of the sensor community towards MoS_2_ and its dopants as promising sensor materials in detecting various environmental gases.^3^ Gases like NH_3_, SO_2_, NO_2_, and H_2_S are to be found in our environment and are generated by naturally occurring processes or human activities on earth. Ammonia is the most prominent among the aforementioned gases. However, ammonia is very useful in areas like the agricultural sector and other research-related activities, but its adverse effect on the environment cannot be overemphasized.^4,5^ From the literature, it has been proven that various health-related challenges like irritation in the respiratory tract and eyes, which may even lead to blindness and death in a few cases, can be caused by long-term exposure to even a small amount of ammonia.^6,7^ Hence, various health agencies worldwide have fixed the maximum limit of ammonia in workplaces at 25 ppm.^8^ Though it is a challenging task to achieve gas sensing under extreme environmental conditions, molybdenum disulfide (MoS_2_), as a typical transition metal with its characteristic of higher charge carrier mobility, has offered us a great opportunity to surmount these challenges to some extent.^9,10^

In line with the development of experimental strategies, density functional theory (DFT) has recently been used by many scientists employing theoretical calculations to predict and understand the mechanistic behaviour, sensitivity and conductivity of the gas sensing ability of many materials. Enhancing the response of NH_3_ graphene-sensors by using devices with different graphene–substrate distances was conducted by Cadore A. R. *et al.*^11^ and their results show that graphene–ammonia gas sensors based on a G/hBN heterostructure exhibit the fastest recovery times for NH_3_ exposure and are only slightly affected by wet or dry air environments. Similarly, Gurleen Kaur Walia *et al.*^12^ performed first-principles investigation on defect-induced silicene nanoribbons—a superior medium for sensing NH_3_, NO_2_ and NO gas molecules—and their work reveals that the introduction of defects can drastically improve the sensitivity of ASiNRs. The optical fingerprints and electron transport properties of DNA bases adsorbed on monolayer MoS_2_ were studied by Munish Sharma *et al.*,^13^ and their results reveal that electronic transport through conjugate systems allows the clear distinction of one nucleobase from one another. In the same vein, the effect of different covalent bond connections and doping on the transport properties of planar graphene/MoS_2_/graphene heterojunctions was conducted by Wei Li *et al.*^14^ Their research shows that the C–S structure exhibits a smaller p-type Schottky barrier, indicating that it has better transport properties than the other two structures for a gas sensing mechanism for dissolved gases in transformer oil on an Ag–MoS_2_ monolayer. Interestingly, the adsorption behaviour of an Rh-doped MoS_2_ monolayer towards SO_2_, SOF_2_, SO_2_F_2_ based on DFT study was carried out by Gui *et al.*^15^ and coworkers and their results reveal that an Rh–MoS_2_ monolayer had good selectivity and gas sensitivity to SO_2_ and SOF_2_ with chemical adsorption phenomena.

This work is tailored towards subjecting our understanding to a framework of providing accurate knowledge on the conductivity, sensitivity, and selectivity of a 2D monolayer material and its doped atoms in detecting ammonia (NH_3_) gas, which requires a sensor that can precisely detect a minimum quantity of a targeted gas like NH_3_. In this work, we employed higher-level theoretical calculation to provide theoretical insights into the electronic properties of MoS_2_ monolayers and its doped elements (boron, nitrogen, phosphorus and silicon) to explore the promising sensing behaviors of MoS_2_-based gas sensors. Knowledge of the electronic properties of sensor materials is of great importance in analyzing sensor properties. Hence, electronic properties such as frontier molecular orbital analysis of the energy of the HOMO and LUMO were evaluated in detail to provide solid knowledge on the sensitivity and conductivity of the studied material, and natural bond orbital analysis was employed to study intermolecular and intramolecular charge transfer between the surface and the adsorbed gas (NH_3_). The geometric structure was fully evaluated after optimization to investigate the change in the electronic properties before and after the adsorption of NH_3_ gas. The adsorption capacity and sensor mechanism of the MoS_2_ surface and its doped elements are discussed in detail by employing four different functionals, as discussed in the methodology. Recently, understanding the recovery time of a sensor material has been important; hence, we studied the recovery time of the studied materials together with charge separation analysis. The conductivity of a sensor material which is a function of changes in energy between the HOMO and the LUMO was investigated and is presented in this work alongside the charge transfer analysis. The interatomic interaction of the studied systems and the nature of the interaction between these MoS_2_ doped surfaces and NH_3_ gas were also characterized by Bader's quantum theory of atoms in molecules (QTAIM) and noncovalent interactions, respectively. Similarly, the electronic transport properties were also evaluated. With these objectives, we very much believe that this study will significantly contribute towards the development of a novel sensor material with much higher conductivity than existing ones.

### 2. Computational calculation details

Theoretical calculations performed on the studied surface of an MoS_2_ monolayer and its doped atoms B@MoS_2_-QD, N@MoS_2_-QD, P@MoS_2_-QD and Si@MoS_2_-QD were carried out with the help of the GaussView 6.0.16 and Gaussian 16 suite of programs.^16,17^ Geometry minimization and energy calculations were carried out by employing the hybrid long-range separated empirical-corrected dispersion (ωB97X-D).^18^ All the systems studied here were calculated in a vacuum using the genECP method by assigning the 6-311++G(d,p) and the LanL2DZ basis sets to the lighter and heavier atoms, respectively. Geometric parameters, including all the bond lengths before and after interaction, were obtained with the help of Chemcraft 1.6 (ref. 19) to study the changes in the bond length and bond strength of the doped surfaces before and after adsorption, since bond length is one of the key factors in understanding the adsorption behaviour of sensor materials. Understanding the electronic distribution and sensor properties is an important concept in sensor studies, so frontier molecular orbital analysis was performed using the log files generated from the geometric optimization from which further calculation using Koopman's approximation was done and is presented in Table S1 of the ESI.† At the same level of theory, using the integrated NBO 3.0 (ref. 20) available in Gaussian 16, natural population analysis was carried out to investigate the charge delocalization and the intermolecular interaction between the adsorbent and the adsorbate. Quantum theory of atoms in molecules (QTAIM) and noncovalent interactions were the topological analyses used to gain more insight into the deeper nature of interatomic interactions and to improve reliability in predicting noncovalent interactions.^21,22^ The computations of QTAIM and NCI were done *via* the Multiwfn 3.7 program developed by Tian Lu *et al.*^23^ Density of states (DOS) analysis was performed for reasons: first to understand the electronic distribution and, secondly, to view the fragment with the most intense contribution to the interactions between the surface and the adsorbate using Guass Sum 3.0 and Multiwfn 3.7, respectively. The HOMO–LUMO plots presented in Table 3 were obtained from Avogadro software.^24^

To fully investigate the adsorption behaviour of NH_3_ on the surface of MoS_2_ and its doped metals, adsorption benchmarking was carried out using single-point energy calculation by employing four different functionals. The M06-2X meta-generalised gradient approximation (GGA) functional exchange;^25^ PBE0 (Perdew–Burke–Ernzerhof exchange);^26^ B3LYP, which consists of the three parameters of Lee–Yang–Parr with the gd3bj dispersion correction;^27^ and ωB97X-D (hybrid long-range separated empirical-corrected dispersion, ωB97X-D functional)^28^ were employed for a benchmarking study to understand and to gain a clear insight into which functional best describes the adsorption mechanism of NH_3_ on the monolayer of MoS_2_ and its doped elements. The results of adsorption energy presented in Table 1 were obtained *via* eqn (1)–(5).

1 *E*_Ad(B@MoS_2_-QD-NH_3_)_ = *E*_B@MoS_2_-QD-NH_3__ − (*E*_B@MoS_2_-QD_ + *E*_NH_3__)

2 *E*_Ad(N@MoS_2_-QD-NH_3_)_ = *E*_N@MoS_2_-QD-NH_3__ − (*E*_N@MoS_2_-QD_ + *E*_NH_3__)

3 *E*_Ad(P@MoS_2_-QD-NH_3_)_ = *E*_P@MoS_2_-QD-NH_3__ − (*E*_P@MoS_2_-QD_ + *E*_NH_3__)

4 *E*_Ad(Si@MoS_2_-QD-NH_3_)_ = *E*_Si@MoS_2_-QD-NH_3__ − (*E*_Si@MoS_2_-QD_ + *E*_NH_3__)

5 *E*_Ad(S@MoS_2_-QD-NH_3_)_ = *E*_S@MoS_2_-QD-NH_3__ − (*E*_S@MoS_2_-QD_ + *E*_NH_3__)

**Table 1:** Selected bond lengths surrounding the doped metals of the studied systems estimated with the ωB97XD/6-311++G(d,p) basis set

System	Bond label	Bond length (Å)	
		Before ads	After ads
B@MoS_2_-QD-NH_3_	B_36_–Mo_13_	2.185	2.243
	B_36_–Mo_4_	1.851	2.109
	B_36_–Mo_15_	2.185	2.213
	B_40_–N_38_	—	1.547
N@MoS_2_-QD-NH_3_	N_36_–Mo_4_	1.891	2.089
	N_36_–Mo_13_	2.031	2.112
	N_36_–Mo_15_	2.031	2.108
	N_40_–N_37_	—	1.419
P@MoS_2_-QD-NH_3_	P_36_–Mo_4_	2.437	2.439
	P_36_–Mo_13_	2.437	2.450
	P_36_–Mo_15_	2.422	2.400
	P_36_–N_33_	—	3.022
Si@MoS_2_-QD-NH_3_	Si_36_–Mo_4_	2.412	2.396
	Si_36_–Mo_13_	2.384	2.399
	Si_36_–Mo_15_	2.412	2.395
	Si_36_–N_38_	—	1.864
S@MoS_2_-QD-NH_3_	S_25_–Mo_15_	2.405	2.405

All other adsorption mechanisms exploited in this study were strictly based on calculations using mathematical equations.

## 3. Results and discussion

### 3.1 Geometric optimization

The optimized structures of the MoS_2_ monolayer and its doped surface, as well as the absorbate which is (NH_3_) gas, are displayed in Fig. 1 and their bond lengths are presented in Table 1. The monolayer of MoS_2_, which is purely made of a honeycomb sheet of molybdenum atoms that are covalently sandwiched between two honeycomb sheets of sulfur atoms, is known to have a hexagonal plane of sulfur atoms on either side of a hexagonal plane of Mo atoms.^29,30^ After geometric optimization using the ωB97XD/6-311++G(d,p) level of theory, the geometrically optimized lattice parameters for the monolayer surface and its dopant before adsorption were observed to have the following bond lengths. For the boron-doped surface (B@MoS_2_-QD) the B_36_–Mo_13_, B_36_–Mo_4_ and B_36_–Mo_15_ bond lengths were 2.185 Å, 1.851 Å and 2.185 Å, respectively. For the N-doped (N@MoS_2_-QD) surface the following bond lengths 1.891 Å, 2.031 Å and 2.031 Å corresponded to N_36_–Mo_13_, N_36_–Mo_4_ and N_36_–Mo_15_, respectively. Similarly, the bond lengths within the P-doped surface (P@MoS_2_-QD) before adsorption were observed to be 2.437 Å, 2.437 Å and 2.422 Å for the following bonds P_36_–Mo_4_, P_36_–Mo_13_ and P_36_–Mo_15_. The (Si@MoS_2_-QD)-doped surface was observed to have lengths of 2.412 Å, 2.384 Å and 2.412 Å for the following bonds surrounding the doped metal Si_36_–Mo_4_, Si_36_–Mo_13_ and Si_36_–Mo_15_, respectively. The bare surface MoS_2_ was observed to have a bond length between molybdenum and sulfur atoms of 2.405 Å. These results are presented in Fig. 1 and Table 1 and show that the (P@MoS_2_-QD)-doped structure had the longest bond length compared to the other doped surfaces.

**Fig. 1:** Optimized structures of MoS_2_ monolayer and its doped (B, N, P, and Si) surface showing the different bond lengths between the doped metal and the surrounding atoms estimated with the DFT/ωB97XD/6-311++G (d,p) basis set.

From Fig. 1, it can be observed that the doped atoms boron, nitrogen, phosphorus, and silicon on the bare surface of MoS_2_ have an effect on its geometrical bond lengths: for example, elongation of MoS_2_ monolayer bonds. Fig. 2 presents the structure of the systems after interaction and the values are also presented as part of Table 1. It is observed that there is an increase in the bond length of the doped surfaces after interacting with NH_3_. The B@MoS_2_-QD-NH_3_ bond length after adsorption increased from 2.185 Å, 1.851 Å and 2.185 Å to 2.243 Å, 2.109 Å and 2.213 Å for B_36_–Mo_13_, B_36_–Mo_4_, and B_36_–Mo_15_, respectively, and the adsorption bond length of Bo_40_–N_38_ was 1.547 Å. The N@MoS_2_-QD-NH_3_ bond length increased from 1.891 Å, 2.013 Å and 2.013 Å to 2.089 Å, 2.112 Å and 2.108 Å for N_36_–Mo_4_, N_36_–Mo_13_, and N_36_–Mo_15_, respectively, and the adsorption bond length of N_40_–N_37_ was 1.419 Å. Similarly, an increase in bond distance was observed in the adsorption of P@MoS_2_-QD-NH_3_ from 2.437 Å, 2.437 Å and 2.422 Å to 2.439 Å, 2.450 Å, and 2.400 Å for P_36_–Mo_4_, P_36_–Mo_13_, and P_36_–Mo_15_, respectively, with an adsorption bond length of 3.022 Å for P_36_–N_33_. Also, observable changes in the bond length were observed after adsorption of Si@MoS_2_-QD-NH_3_ which resulted in a change in the bond length from 2.412 Å, 2.384 Å and 2.412 Å to 2.396 Å, 2.399 and Å 2.395 Å for Si_36_–Mo_4_, Si_36_–Mo_13_ and Si_36_–Mo_15_, respectively, with an adsorption bond length of 1.864 Å for S_25_–N_38_. The bond length between the monolayer of MoS_2_ and its complex (interacted surface) was observed to remain unchanged due to the covalent nature of the sandwich atoms. Thus, it is obvious that N@MoS_2_-QD-NH_3_ has the shortest bond length, implying that it is the most stable complex. This could be explained by the higher electronegativity of the doped atoms and hence the higher electronegativity compared to the other dopants.

**Fig. 2:** Optimized structures of MoS_2_ monolayer and its doped atoms (B, N, P, and Si) interacting with a molecule of NH_3_ gas, indicating the different bond lengths surrounding the doped metals estimated with the DFT/ωB97XD/6-311++G(d,p) basis set.

### 3.2 HOMO–LUMO analysis

Understanding the sensing characteristics and the conductivity of a sensor material is very crucial to the sensor community since it determines the working principle of a constructed gas sensor material. Owing to this, frontier molecular orbital (FMO) analysis, which plays an exceptional role in the computational design of sensors, was carried out in this study. This analysis consists of the highest occupied molecular orbital (HOMO) and the lowest unoccupied molecular orbital (LUMO).^31^ Information about the sensing abilities of the free sensor materials and complexes can be obtained from the difference between the relative energies of the HOMO and LUMO.^32,33^ The HOMO–LUMO plots of the materials under study are presented in Fig. 3 and their energies are given in Table 2. The bare surface of the monolayer of MoS_2_ was observed to have an energy gap of 3.3105 eV. After doping the surface with boron, nitrogen, phosphorus and silicon atoms, the energies of HOMO, LUMO and their differences were observed to increase, which could be explained based on the periodic characteristics in the doped atoms.^32,33^ Before interaction of the doped surface with NH_3_, the HOMO and LUMO values of B@MoS_2_-QD were −9.8067 eV and −6.4450 eV, respectively, with a band gap of 3.3617 eV. After interaction, the adsorption of NH_3_ on the surface of B@MoS_2_ caused an increase in the HOMO–LUMO values of B@MoS_2_-NH_3_ to −9.8336 eV and −5.8753 eV, respectively, leading to an increase in the band gap from 3.3617 eV to 3.9583 eV, as presented in Table 2.

**Fig. 3:** Pictorial display of HOMO–LUMO analysis.

**Table 2:** HOMO, LUMO, band gap and Fermi-level energies of the studied systems theoretically calculated at different levels of theory

Functionals	Surfaces	HOMO/eV	LUMO/eV	Band gap/eV	*E*_FL_
ωB97XD	B@MoS_2_-QD	−9.8067	−6.4450	3.3617	8.1259
	N@MoS_2_-QD	−9.7017	−6.3261	3.3756	8.0139
	P@MoS_2_-QD	−9.6369	−6.2986	3.3383	7.9678
	Si@MoS_2_-QD	−7.9806	−3.6357	4.3448	5.8081
	MoS_2_	−7.1952	−3.8847	3.3105	5.5400
	B@MoS_2_-NH_3_	−9.8336	−5.8753	3.9583	7.8544
	S@MoS_2_-NH_3_	−7.4605	−3.4626	3.9979	5.4615
	Si@MoS_2_-NH_3_	−7.7089	−3.2465	4.4624	5.4777
	N@MoS_2_-NH_3_	−10.4652	−5.8765	4.5887	8.1692
	P@MoS_2_-NH_3_	−9.7658	−5.8548	3.911	7.8103
PBE1PBE	B@MoS_2_-NH_3_	−8.3862	−7.2420	1.1442	7.8141
	N@MoS_2_-NH_3_	−8.9253	−7.3062	1.6191	8.1157
	P@MoS_2_-NH_3_	−8.7699	−7.7859	0.984	8.2779
	Si@MoS_2_-NH_3_	−5.8626	−4.9701	0.8925	5.4163
	S@MoS_2_-NH_3_	−5.9628	−4.8150	1.1478	5.3889
B3LYP	B@MoS_2_-NH_3_	−8.2181	−7.2858	0.9323	7.7519
	N@MoS_2_-NH_3_	−8.7013	−7.3625	1.3388	8.0319
	Si@MoS_2_-NH_3_	−5.7203	−5.0120	0.7083	5.3661
	S@MoS_2_-NH_3_	−5.7995	−4.8591	0.9404	5.3293
M06-2X	B@MoS_2_-NH_3_	−9.2578	−6.6131	2.6447	7.9354
	N@MoS_2_-NH_3_	−9.8328	−6.7269	3.1059	8.2798
	P@MoS_2_-NH_3_	−9.5484	−7.3470	2.2014	8.4477
	Si@MoS_2_-NH_3_	−6.5753	−4.4528	2.1125	5.5140
	S@MoS_2_-NH_3_	−6.8795	−4.1554	2.7241	5.5174

Using DFT/ωB97XD/6-311++G(d,p), the energy gap before adsorption was observed to follow the trend MoS_2_ < P@MoS_2_-QD < B@MoS_2_-QD < N@MoS_2_-QD < Si@MoS_2_-QD, with corresponding energy gaps of 3.3103 eV, 3.3383 eV, 3.3617 eV, 3.3756 eV and 4.3448 eV, respectively. As was observed in the case of adsorption of NH_3_ gas on B@MoS_2_-QD, the adsorption of NH_3_ gas on N@MoS_2_-NH_3_, S@MoS_2_-NH_3_, and P@MoS_2_-NH_3_ similarly causes an increase in the band gap as follows: 4.5887 eV (N@MoS_2_-NH_3_), 3.9979 eV (S@MoS_2_-NH_3_) and 3.911 eV (P@MoS_2_-NH_3_), and this increase in the band gap is a result of an increase in the HOMO–LUMO values after interaction. It was also observed that the functionalization of the interactions with the doped surface on adsorption of NH_3_ brought about a total decrease in the difference between the conduction band and the valence band, indicating an increase in conductivity of the gas towards the surface, as has been reported in other adsorption studies.^34^ With the PBE1PBE functional the adsorption of NH_3_ on the surfaces of the complexes results in a decrease in the HOMO–LUMO values, which also decreases the band gap. As presented in Table 2, the PBE1PBE functional gives the lowest energy gap compared to the other functionals, indicating the higher conductivity and sensitivity of the adsorbate on the surfaces of MoS_2_ and its doped metals. From Fig. 3, one can observe that the delocalization of the electronic cloud arising from the difference in the conduction and the valence band resulted in increased conductivity of the studied sensor materials, as observed. Thus, for the B@MoS_2_-NH_3_ complex, the HOMO was highly delocalized on the Mo atoms of the MoS_2_ surface and on some part of the boron-doped atom while the LUMO was only concentrated on the Mo atoms of the surface. Similarly, for the N@MoS_2_-NH_3_, delocalization of the electron cloud from HOMO was on the sulfur atoms and a little part of it was on the Mo atoms of the surface. From the LUMO orbital the nitrogen-doped atom and part of the Mo atoms were highly concentrated with electrons. For the P@MoS_2_-NH_3_ complex, the electron delocalization for both HOMO and LUMO was not concentrated on the doped phosphorus atom but concentrated on the Mo atoms, particularly for the LUMO. In the Si@MoS_2_-NH_3_ complex, the HOMO was highly concentrated on the Mo and S atoms that made the monolayer of MoS_2_ and the Si-doped complex seem to be unoccupied by the electron cloud. While the LUMO was highly concentrated on the Si-doped atoms on the surface of MoS_2_, part of the absorbate was also observed to have an electron cloud. For the interaction of the bare MoS_2_-NH_3_ the HOMO was highly concentrated on the covalent atoms of Mo and S atoms that formed the surface and the LUMO was mostly on the Mo atoms.

The sensitivity and conductivity of the studied sensor material were further studied and analyzed by invoking the popular Koopmans approximation.^35^ Quantum chemical indicators were used, such as chemical hardness (*η*), which is described as the resistance of atoms or atom groups to charge transfer;^36^ electronegativity (*χ*), the tendency of an atom or atom group to attract electrons;^37^ chemical potential (*μ*) or electronic potential, the measure of the likelihood of an atom or group of atoms to escape its ground/non-excited state;^38^ electrophilicity index (*ω*), a measure of the electron acceptor affinity to gain an additional electronic charge from the surrounding systems;^39^ and chemical softness (*σ*), which correctly describes the tendency of an atom to receive electron/electrons.^40^ These parameters provide more elucidation into the reactivity, chemical stability, and intermolecular interactions, as well as the electric and optical properties of the titled systems, which were estimated using Koopmans' approximation and conceptual density theory. These parameters were vividly studied, and the results are presented in Table S1 of the ESI† for a clearer understanding and affirmation of the gas sensing characteristic such as conductivity, gas sensitivity and electronic properties of the surface, such as the chemical reactivity and stability of the adsorbent and the adsorbate.

The TDOS plot presented in Fig. 4, was used to further predict the changes in the electronic energy of the studied gas sensor systems B@MoS_2_-NH_3_, N@MoS_2_-NH_3_, P@MoS_2_-NH_3_, Si@MoS_2_-NH_3_ and MoS_2_-NH_3_ calculated at the ωB97XD/6-311G++(d,p) level and plotted with the help of the Gauss sum package, as mentioned in computational methods. The plots display the electronic properties of the occupied and the virtual orbitals alongside the energy gaps of the studied interacted surfaces. These plots were comparably plotted to provide better insight into the difference arising between the occupied orbital and the virtual orbital due to the interaction between the adsorbent and the adsorbate. The changes in the TDOS peak intensities, as well as the peak shifts, are indications of the changes in the transition of electrons from the occupied orbital to the virtual orbitals, reflecting the changes in conductivity upon the adsorption of NH_3_ on the surface of MoS_2_ and its doped metal complexes.^41^ From Fig. 4 it can be observed that more prominent changes in the TDOS peak intensities and energy level were observed in the occupied orbitals of the complex. This was observed to be in agreement with the frontier molecular orbital analysis, in that the highest change in the energy gap of P@MoS_2_-NH_3_ is observed due to significant changes in the HOMO energy level.

**Fig. 4:** Density of states (DOS) plots for B@MoS_2_-NH_3_, N@MoS_2_-NH_3_, P@MoS_2_-NH_3_Si@MoS_2_-NH_3_ and MoS_2_-NH_3_ calculated at the ωB97XD/6-311G++(d,p) level of theory.

### 3.3 Analysis of natural bond orbital

To obtain deeper insight into the sensing mechanism, conductivity and the transfer of electrons from the doped surfaces of B@MoS_2_-QD, N@MoS_2_-QD, P@MoS_2_-QD, Si@MoS_2_-QD and S@MoS_2_-QD and the adsorbate (NH_3_) gas, natural bond orbital analysis, which studies the intermolecular and intramolecular charge transfer resulting in an understanding of the bonding concept, was carried out on the studied systems. Insight into intramolecular and intermolecular hyper-conjugation, electron delocalization, and intermolecular charge transfer (ICT) with the donor and acceptor occupancy, hybrid, and atomic orbital persisting within the studied surfaces were obtained by employing the ωB97XD/6-311++G(d,p) level of theory. The nature of the interaction existing between the donor orbital and acceptor orbital is expressed in terms of second-order perturbation energy (*E*^(2)^) or stabilization energy (*E*^(2)^).^42^ A thorough literature review showed that the higher the stabilization energy the stronger the interaction between the donor orbital and acceptor orbital and the stronger the strength of adsorption of the sensing materials.^43^ The second-order perturbation energy of the studied doped MoS_2_ monolayer and its interaction with NH_3_ gas was estimated using eqn (6) ^44^6where *q*_*i*_ is the donor orbital occupancy, *ε*_*i*,_ and *ε*_*j*_ represent the diagonal elements and *F*_(*i*,*j*)_ stands for the off-diagonal elements of the Fock matrix.

The estimated second-order perturbation of the MoS_2_ monolayer and its doped surface before and after adsorption resulting in the higher delocalization of the whole system are presented in Table 3. Detailed information about the natural bond orbital analysis is presented in Table S2 of the ESI† for clear insight into the analysis. From this study different transitions were observed to occur in the different surfaces due to the differences in the size and electronegativity of the doped atoms. From Table 3 it was observed that before adsorption of the NH_3_ molecule on the doped surfaces, the second-order perturbation energies were in the order B@MoS_2_-QD > Si@MoS_2_-QD > N@MoS_2_-QD > S@MoS_2_-QD > P@MoS_2_-QD corresponding to the respective energies 5389.14 kcal mol^−1^ and 5797.69 kcal mol^−1^ for the boron-doped surface, 1640.59 kcal mol^−1^ and 1044.65 kcal mol^−1^ for the silicon-doped surface, 934.35 kcal mol^−1^ and 966.99 kcal mol^−1^ for the nitrogen-doped surface, 700 kcal mol^−1^ and 621 kcal mol^−1^ for the bare MoS_2_ surface, and the phosphorus-doped MoS_2_ surface was observed to have perturbation energies of 700.05 kcal mol^−1^ and 621.20 kcal mol^−1^. From this the doped surface B@MoS_2_-QD was observed to have the highest perturbation energy resulting from the transitions LP → σ* and π* → σ*, indicating stronger interaction at this doped metal compared to the other doped surfaces. As presented in Table 3, a great decrease in the perturbation energies was observed after adsorption of the molecule of NH_3_ on the surface of the doped MoS_2_ monolayer, indicating the stability of the adsorbate on the MoS_2_ doped surfaces. From the obtained results presented here in Table 3, the most persistent form of donor–acceptor orbital interaction resulting from intermolecular hyper-conjugation existing within the studied surface and its doped atoms was observed to have ten different transitions: LP* → σ*, π* → σ*, σ* → σ*, σ → σ, LP* → LP*, π* → π*, LP → LP*, π* → σ*, σ* → LP, and LP* → σ*.

**Table 3:** Donor (*i*), occupancy, acceptor (*j*), stabilization energies, hybrid orbital and atomic orbital of the studied systems

Surface	Donor (*i*)	Occupancy	Acceptor (*j*)	Occupancy	*E* ^(2)^/kcal mol^−1^	*E*(*j*) − *E*(*i*)	*F*(*j*, *i*)	Hybrid	Atomic orbital
B@MoS_2_-QD	LP(1) Mo_15_	0.41943	σ*Mo_5_–Mo_15_	0.46915	5389.14	0.02	0.443	spd^69.55%^	s (7.61%) p (33.11%) d (59.28%)
	π*Mo_4_–Mo_5_	0.41190	σ*Mo_5_–Mo_15_	0.46915	5797.69	0.03	0.553	spd^66.59%^	s (8.60%) p (2.80%) d (88.60%)
N@MoS_2_-QD	σ*M0_5_–S_24_	0.19917	σ*Mo_5_–Mo_15_	0.35611	934.35	0.02	0.215	spd^50.76%^	s (25.11%) p (15.35%) d (59.54%)
	σMo_8_–Mo_13_	0.31210	σMo_8_–Mo_14_	0.27945	966.99	0.07	0.254	spd^72.00%^	s (13.49%) p (0.90%) d (85.61)
P@MoS_2_-QD	σ*Mo_1_–Mo_13_	0.37352	σ*Mo_1_–S_3_	0.15584	583.69	0.02	0.193	spd^57.74%^	s (16.41%) p (13.56%) d (70.03%)
	LP*Mo_16_	0.38276	LP*Mo_14_	0.36994	655.03	0.02	0.149	spd	s (13.52%) p(78.27%) d(8.21%)
Si@MoS_2_-QD	π*Mo_14_–S_30_	0.19163	π*Mo_14_–S_23_	0.16096	1640.59	0.03	0.273	spd^64.82%^	s (14.91%) p (36.06%) d (49.03%)
	LP Si_36_	0.21354	LP*(2) Mo_13_	0.30269	1044.65	0.05	0.331	spd	s (0.12%) p (91.39%) d(8.49%)
MoS_2_-QD	LP*(3) Mo_4_	0.34154	LP* Mo_13_	0.38483	700.05	0.01	0.143	spd	s (0.05%) p (87.20%) d (12.75%)
	πMo_1_–Mo_8_	0.65040	σ*Mo_1_–Mo_8_	0.36176	621.20	0.09	0.257	spd^50.00%^	s (14.17%) p (24.84%) d (60.98%)
B@MoS_2_-NH_3_	LP*(2) Mo_16_	0.34380	LP*(2) Mo_5_	0.10959	4107.17	0.02	0.508	spd	s (0.91%) p (92.76%) d (6.34%)
	σ*Mo_8_–Mo_14_	0.59437	σ*Mo_8_–S_9_	0.27539	1353.59	0.02	0.221	spd^33.17%^	s (13.62%) p (25.15%) d (61.23%)
N@MoS_2_-NH_3_	σ*Mo_8_–S_11_	0.28146	σ*Mo_8_–S_9_	0.24751	1892.76	0.02	0.312	spd^62.86%^	s (25.54%) p (7.38%) d (67.08%)
	σ*Mo_8_–S_11_	0.28146	LP*Mo_14_	0.35384	1091.40	0.02	0.198	spd	s (0.90%) p (89.95%) d (9.15%)
P@MoS_2_-NH_3_	LP Mo_16_	0.38509	LP*Mo_15_	0.36750	1012.07	0.02	0.201	spd	s (10.22%) p (80.47%) d (9.32%)
	σMo_8_–S_9_	1.81052	πMo_1_–S_9_	1.86390	774.80	0.15	0.346	spd^41.87%^	s (12.41%) p (10.15%) d (77.44%)
Si@MoS_2_-NH_3_	σ*Mo_20_–S_28_	0.39827	LPMo_20_	0.40970	645.69	0.04	0.216	spd	s (8.84%) p (65.52%) d (25.64%)
	σ*Mo_18_–S_34_	0.18666	σ*Mo_18_–S_24_	0.32422	418.95	0.02	0.177	spd^62.61%^	s (16.58%) p (8.07%) d (75.36%)
S@MoS_2_-NH_3_	LP* Mo_13_	0.35435	LP*(2) Mo_1_	0.11457	477.23	0.01	0.132	spd	s (1.29%) p (90.54%) d (8.18%)
	LP* Mo_8_	0.17664	σ*Mo_8_–S_11_	0.25851	449.27	0.01	0.133	spd^59.26%^	s (8.61%) p (21.06%) d (70.33%)

From the displayed second-order perturbation energy *E*^(2)^ of the studied complexes, an inverse relationship exists between the perturbation energies and the FMO studies, in that the doped surface with the lowest energy gap tends to have an increased perturbation energy after adsorption of NH_3_ gas on the surface. It worth mentioning that adsorption of NH_3_ molecules on the doped surface brought about a decrease in perturbation energies for the boron-doped, silicon-doped and bare surfaces, indicating the stability of the surfaces; but for the phosphorus-doped and nitrogen-doped surfaces an increase in the perturbation energy was observed, indicating an increase in conductivity of the studied systems. The higher perturbation energies observed after interaction, as displayed in Table 3, were 4107.17 kcal mol^−1^ and 1353.59 kcal mol^−1^ for B@MoS_2_-NH_3_, 1892 kcal mol^−1^ and 1091.40 kcal mol^−1^ for N@MoS_2_-NH_3_, 1012.07 kcal mol^−1^ and 774.80 for P@MoS_2_-NH_3_, and 645.69 kcal mol^−1^ and 418.95 kcal mol^−1^ for Si@MoS_2_-NH_3_. Similarly, higher perturbation energies of 477.23 kcal mol^−1^ and 449.27 kcal mol^−1^ were observed for the bare surface of the MoS_2_ monolayer. The occupancy values for donor and acceptor orbitals as well as the hybrid orbital and the atomic orbital of the studied systems have been carefully studied and are presented in Table 3. The delocalization of the π system within the studied surface was also evaluated using occupancy of the Lewis donor, and the acceptor of P@MoS_2_-NH_3_ was observed to have the highest occupancy that corresponded to its lowest energy gap. For the atomic orbital contribution, it was observed that (σMo_8_–Mo_14_) from the nitrogen-doped atom interaction on the NH_3_ had the major percentage of spd at 72.00%, arising from the atomic contributions of s (13.49%), p (0.90%) and d (85.61) compared to other sensing materials.

### 3.4 Comparative adsorption studies

The sensing ability of MoS_2_ and its doped atoms was also investigated by calculating the adsorption energy between the adsorbent and the adsorbate by carrying out a comparative adsorption study using M062-X, ωB97XD, B3LYP, and PBE0 within the framework of density functional theory at 6-311G ++(d,p) level. In order to investigate the adsorption energy of the complex and its behavior in various functionals and the mechanism of the adsorption energy by climbing the Jacob's ladder of functionals, the adsorption energy was calculated in the gas phase using eqn (1)–(5), as mentioned in Section 2 and the calculated results are displayed in Table 4. As can be seen in Table 4, the *E*_ad_ values obtained showed a relatively stable conformation and strong interaction, although more negative values were obtained from ωB97XD, indicating an exothermic reaction and a chemical adsorption interface. From this analysis, P@MoS_2_-NH_3_ was observed to have the strongest interaction between its phosphorus-doped MoS_2_ surface and NH_3_ due to its higher negative adsorption energy which is an indication of chemical adsorption, which further indicates the better adsorbing potential for the adsorbate.^45^ Weak adsorption of NH_3_ on the surface of MoS_2_ and its doped surface was observed with the functionalization of the systems P@MoS_2_-NH_3_ and Si@MoS_2_-NH_3_, as can be seen from Table 4, indicating physical adsorption as a well an endothermic reaction.^46^ The adsorption energies of the doped metals B, N, P, Si and the bare surface of MoS_2_ in the four functionals were observed to decrease due to the interaction between the metal atoms and bare MoS_2_. The adsorption energies of B@MoS_2_-NH_3_ were observed to be −1.838, −1.732, −1.9058 and −5.759, corresponding to the functionals ωB97XD, rpbe1pbe, B3LYP and M06-2X, respectively. N@MoS_2_-NH_3_ was observed to have adsorption energies of −5.872, −4.939, −4.3875 and −1.8046 with the ωB97XD, PBE1PBE, B3LYP and M06-2X functionals, respectively.

**Table 4:** Comparative adsorption studies employing four different functionals using ωB97XD, PBE1PBE, B3LYP and M06-2X with the 6-311++G(d,p) basis set

System	ωB97XD	PBE1PBE	B3LYP	M06-2X
B@MoS_2_-NH_3_	−1.838	−1.732	−1.9058	−5.759
N@MoS_2_-NH_3_	−5.872	−4.939	−4.3875	−1.8046
P@MoS_2_-NH_3_	−75.191	7.120	8.047	6.403
Si@MoS_2_-NH_3_	−3.038	6.638	6.646	6.643
S@MoS_2_	−17.170	−0.224	−1.841	−0.761

P@MoS_2_-NH_3_ also had an adsorption energy of −75.191 with ωB97XD and positive adsorption energies of 7.120, 8.047 and 6.403, indicating an endothermic reaction could be observed for PBE1PBE, B3LYP and M06-2X, respectively. Similarly, Si@MoS_2_-NH_3_ was also seen to have positive adsorption energies with pbe1pbe, B3LYP and M06-2X, and a negative value of −3.078 was observed with the ωB97XD functional. The bare surface of MoS_2_ was observed to have the adsorption energies −17.170, −0.224, −1.841 and −0.761 for the functionals ωB97XD, PBE1PBE, B3LYP and M06-2X, respectively. From the adsorption benchmarking, ωB97XD was observed to have the highest negative values, indicating stronger and better adsorbing potential for the adsorbate (NH_3_) than all the other functionals used, and it is important to note that P@MoS_2_-NH_3_ with the highest negative value (−75.191 kcal mol^−1^) has better adsorbing potential for detecting the gas (NH_3_). This characteristic observed here for the phosphorus-doped MoS_2_ monolayer was also observed from the frontier molecular analysis, as the surface had the lowest gap between the conduction and the valence bands. P@MoS_2__NH_3_ was also observed from the quantum theory of atoms in molecules to have the highest Laplacian of electron density (of 0.5809 a.u.) indicating stronger interaction corresponding to previously reported work.^47^

### 3.5 Sensor mechanisms

Sensor mechanisms, such as recovery time, dipole moment, work function, the natural charge before and after adsorption, and change in the charge transfer and conductivity between the adsorbate and the adsorbent, have been used in this study to better understand the conductivity, sensitivity and electronic properties of the studied materials in order to understand the mechanism of the gas sensing ability of the studied surfaces.^48^

#### 3.5.1 Dipole moment and recovery time

To gain more insight into the charge separation within the studied sensor material, information on dipole moment is efficiently used, since it allows one to gain more knowledge into the charge separation within the studied system. With information on the dipole moment, the strength of interaction for studied complexes can be predicted.^49^ Using the ωB97X-D functional, we calculated the dipole moment for all studied systems in the gas state. The magnitude of the charge and the distance between the centers of the positive and negative charges in a system can be related to the distance between the absorbate and the adsorbent. From this study, the bare surface MoS_2_–NH_3_ was observed to have the least dipole moment of 0.0201. From the result obtained after doping, the dipole moment was observed to increase significantly based on the charge separation in the doped atoms. The dipole moments of the doped surface were observed to be 2.3130, 1.6962, 1.5659, and 3.3927 for B@MoS_2_-NH_3_, N@MoS_2_-NH_3_, P@MoS_2_-NH_3_ and Si@MoS_2_-NH_3_, respectively, indicating the higher charge separation and stronger interaction of the Si@MoS_2_-NH_3_ complex. Calculating the recovery time of a sensor material is very essential to the sensor community since it reflects the stability and reusability of the sensor material. Experimentally, the recovery time of a sensor is calculated by applying thermal and electric field effects.^50^ This concept can be theoretically calculated by employing the transition state theory, as shown in eqn (7):^51^7where *τ*, *V*, *E*_ad_, *K* and *T* stand for the recovery time, attempt frequency, adsorption energy, Boltzmann constant and temperature, respectively. From the literature, it has been found that the higher the magnitude of the negative of *E*_ad_, the longer the recovery time.^52,53^ Hence in this study a higher negative adsorption energy was observed for P@MoS_2__NH_3_, which shows it could be useful as a sensor material.

#### 3.5.2 Conductivity and charge transfer

The conductivity of a sensor material is a function of the difference in energy between the highest occupied molecular orbital and the lowest unoccupied molecular orbital.^54^ A literature review shows that a decrease in the energy between the conduction band and the valence bond is an indication of an increase in conductivity of such a sensor material. Hence the electrical conductivity of a sensor material depends on its ability to move electrons from the valence band to the conduction band.^55^ The variations in the electronic characteristics of bare MoS_2_ and its doped atoms may cause changes in the electrical conductivity and resistivity, which can be theoretically calculated using eqn (8):^56^

8 *σ* = *AT*^2/3^exp(*E*_g_/2*KT*)

where the electrical conductivity, constant, temperature, and Boltzmann constant are designated by *σ*, *A*, *T* and *K*, respectively. The sensing response is computed based on the formula:^57^

9 *S* = |*R*_2_ − *R*_1_|/*R*_1_ = |*R*_2_/*R*_1_| − 1

where *R*_1_ and *R*_2_ designate the resistivity of MoS_2_ and its doped atoms after interacting with the NH_3_ molecule. There is an inverse relation between resistivity and electrical conductivity.

The electronic charge transfer between the adsorbate and the adsorbent was also investigated using the natural charge on the MoS_2_ surface and its doped atoms before and after interaction, and the results are presented in Table 5. This is very essential in analysis of the charge transfer between the surface and NH_3_ gas. From the ∇_QNBO_ result, the following differences in the charge were observed: −0.3226, −0.6338, −0.1530, 0.3795 and 0.0088 corresponding to B@MoS_2_-NH_3_, N@MoS_2_-NH_3_, P@MoS_2_-NH_3_, Si@MoS_2_-NH_3_, and MoS_2_-NH_3_, respectively. The higher value of 0.03795 for Si@MoS_2__NH_3_ is an indication of the strong charge transfer between the surface and the adsorbate.

**Table 5:** Dipole moment, natural charge on the adsorbent before and after interaction and work function (*Φ*) of the studied systems estimated with DFT/ωB97XD/6-311++G(d,p)

System	Dipole moment	QNBO before adsorption	QNBO after adsorption	∇_QNBO_	*Φ*
B@MoS_2_-NH_3_	2.3130	1.9978	1.3226	−0.3226	−7.8544
N@MoS_2_-NH_3_	1.6962	−0.7779	−0.1441	−0.6338	−5.4615
P@MoS_2_-NH_3_	1.5659	1.0911	1.24024	−0.1530	−5.4777
Si@MoS_2_-NH_3_	3.3927	2.1466	1.7671	0.3795	−8.1692
MoS_2_-NH_3_	0.0201	0.2245	0.2157	0.0088	−7.8103

### 3.6 Noncovalent interactions

Noncovalent interaction analysis was done at ωB97XD/6-311++G(d,p) basis level to elucidate and vividly quantify the intermolecular and intramolecular interactions between MoS_2_-QD-NH_3_ and the doped atoms (boron, nitrogen, phosphorus and silicon). As a result, NCI differs from covalent bond interaction in that it does not require the exchange of electrons but rather justifies more distributed variations of electromagnetic interactions between molecules or within a molecule.^58^ The different dimensions or categories of noncovalent contact are generally claimed to exist as electrostatic interaction, π effects, van der Waals forces, and hydrophobic effects. Without a doubt, the formation of NCI is studied in terms of the release of chemical energy, which is typically on the scale of 1–5 kcal mol^−1^ (1000–5000 calories per 6.02 × 10^23^ molecules). Computational visualization of intramolecular and intermolecular interactions within and between the complexed molecules revealed several astonishing zones permitted by the isosurfaces created, including van der Waals contacts, steric repulsion, and strong attractions, as can be seen in Fig. 5. The green isosurfaces depict weak interactions due to van der Waals dispersion forces, which seek to explain the fluctuation in charges resulting in a non-specific and non-directional attraction.^59^ The red isosurfaces, on the other hand, depict strong interactions primarily due to steric repulsion, though they influence the conformation and reactivity of ions and molecules. Nevertheless, the scatter maps establish the appearance of peaks in extremely very negative zones of the eigenvalue (*λ*_2_) depicted by the blue color on the horizontal axis, implying that the complexes (S@MoS_2_-QD-NH_3_, Si@MoS_2_-QD-NH_3_, P@MoS_2_-QD-NH_3_, N@MoS_2_-QD-NH_3_, and B@MoS_2_-QD-NH_3_) must have very strong attractive intermolecular interactions, confirming the existence of hydrogen bonds which stabilize the interactions. Instantaneously, peaks at genuine positive zones reflecting the red isosurfaces swiftly corroborate the presence of steric repulsion in all the complexes, thereby triggering destabilizing interactions, consequently complementing the electronic effects, and accounting for the conformation and reactivity of the complexes.^60^ However, van der Waals forces depicted by the green peaks existing between these two regions (strong attractive interaction and steric repulsion) are characterized as regions with low electron density when the eigenvalue (*λ*) approaches zero. On the other hand, this may explain why imperfect fits between interacting complexes are energetically costly, prohibiting association because surface groups tend to interfere. Nonetheless, the complexes revealed van der Waals interactions, resulting in increased energy adsorption and shorter equilibrium distances.

**Fig. 5:** Pictorial representation of the analysis of noncovalent interaction.

When examining these interactions, it is worth noting that the hydrogen bond detected in Si@MoS_2_-QD-NH_3_ is identical to that observed in B@MoS_2_-QD-NH_3_, indicating a stronger interaction because the virtual RDG isosurfaces have a deep blue color. Indeed, compared to Si@MoS_2_-QD-NH_3_ and B@MoS_2_-QD-NH_3_, the 3D RDG isosurfaces clarifying the intermolecular hydrogen bond interaction of S@MoS_2_-QD-NH_3_, B@MoS_2_-QD-NH_3_, and P@MoS_2_-QD-NH_3_ are somewhat green, making such a connection particularly unstable. Furthermore, within the five complexes, the depth of the blue color bonded by the RDG isosurfaces and the accompanying spike peaks are very similar, indicating strong hydrogen bond interaction, as the spike peaks range from approximately 0.00 to 1.40 a.u. In conclusion, it appears difficult to compare the strength of hydrogen bonding between the studied complexes because their respective peaks elucidate only sufficiently strong attractive intermolecular interactions. Thus, it is based on the accuracy of the values integrated over the volume bounded by the RDG surfaces, which is a function of grid spacing.

### 3.7 Bader quantum theory of atoms in molecules (QTAIM)

The topology analysis proposed by Bader, which was first used for analyzing electron densities in “atoms in molecules”, can be applied to any real function and was further employed in this study to evaluate the nature of interaction and bond formation between the doped monolayer of MoS_2_ and its adsorbate NH_3_ using some common real space functions of the topological parameters: density of all electrons *ρ*(*r*), Lagrangian kinetic energy *G*(*r*), Hamiltonian kinetic energy *K*(*r*), potential energy density *H*(*r*), Laplacian of electron density ∇^2^*ρ*(*r*), electron localization function (ELF), energy density *H*(*r*), wave function value for orbitals (*Ψ*_orbital_), ellipticity of electron density (*e*), and eigenvalues of the Hessian (*λ*_1_, *λ*_2_, and *λ*_3_), all estimated at different bond critical points (BCPs) of the studied systems. The highest and the most significant calculated topology parameters in this study are presented in Table 6 for a better understanding of the kinds of bond formation between the adsorbent and the adsorbate and also to gain a clear insight into the sensing ability of the studied materials. A multifunctional wave function analyzer was used in this research for the purpose of studying the noncovalent interactions in the studied systems. Much attention was given to the density of electrons, its Laplacian and the eigenvalues of the Hessian (*λ*_1,_*λ*_2_, and *λ*_3_). Through a literature review it was found that for closed-shell interactions, the values of *ρ*(*r*) vary from 0.002 to 0.016 a.u. for weak van der Waals forces and from 0.0024 to 0.0547 a.u. for strong electrostatic interactions.^61^ For the purpose of this research, the obtained values of *ρ*(*r*) indicated an electrostatic interaction between the doped surface and the gas molecules.^62^ Knowledge of ∇^2^*ρ*(*r*) shows that strong shared-shell interatomic interaction is evidenced by a local concentration of the electron density distribution at the critical point when ∇^2^*ρ*(*r*) < 0; on the other hand, weak closed-shell (CS) interaction exhibits local depletion when ∇^2^*ρ*(*r*) > 0. Greater electron density at bond critical points (BCPs) indicates greater structural stability. Hence an understanding of the stability and reactivity of a sensor material is of significant importance to the sensor community.^63^ Much information about the attractive and repulsive nature of the interaction between the doped surface and the adsorbate (NH_3_) was provided through the second eigenvalue. A literature review shows that a positive value of *λ*_2_ is an indication of steric repulsion, which is a destabilizing interaction, while a negative value indicates an attractive force, which is a stabilizing interaction.^64^

**Table 6:** Calculated Bader values of the Bader theory of atoms in molecules of the studied systems estimated with DFT/ωB97XD/6-311++G (d,p)

Bond	Cp	*ρ*(*r*)	∇^2^*ρ*(*r*)	*G*(*r*)	*K*(*r*)	*V*(*r*)	*H*(*r*)	ELF	*Ψ*_orbital_	*λ*_1_	*λ*_2_	*λ*_3_	*e*
**B@MoS**_**2**_-**NH**_**3**_													
B_40_–N_36_	46	0.1995	0.5787	0.1377	−0.695	−0.1307	0.6946	0.8552	−0.2424	−0.1927	0.9179	−0.1464	0.3160

**N@MoS**_**2**_-**NH**_**3**_													
N_40_–N_37_	68	0.1442	0.5282	0.2477	0.116	−0.3635	−0.1157	0.1746	−0.8710	−0.1253	−0.1394	0.7930	0.1122
Mo_4_–S_3_⋯H_39_	44	0.1731	0.5138	0.1190	−0.9446	−0.1095	0.9446	0.7233	−0.1539	−0.1128	0.7820	−0.1554	0.3776
Mo_5_–S_31_⋯H_38_	64	0.1321	0.4572	0.9796	−0.1634	−0.8162	0.1634	0.4468	−0.3503	0.6324	−0.1061	−0.6909	0.5361

**P@MoS**_**2**_-**NH**_**3**_													
P_36_–N_37_	58	0.1807	0.5809	0.1305	−0.1466	−0.1158	0.1466	0.6956	−0.1717	−0.1323	−0.1300	0.8433	0.0171
Mo_8_–S_11_⋯H_37_	66	0.6711	0.1800	0.5595	0.1096	−0.6692	−0.1096	0.2443	0.5761	−0.5973	0.2953	−0.5550	0.0761
S_3_–N_37_	43	0.9928	0.3006	0.6415	−0.1102	−0.5313	0.1102	0.4031	−0.1476	−0.6212	−0.5097	0.4137	0.2187

**Si@MoS**_**2**_ **–NH**_**3**_													
Si_36_–N_38_	64	0.8034	0.4400	0.4013	0.3948	−0.7962	−0.3948	0.5884	−0.1486	−0.9331	−0.9401	0.6273	0.0074
Mo1–S_3_⋯H_39_	42	0.1435	0.4088	0.9281	−0.9387	−0.8342	0.9387	0.6429	0.2152	−0.1245	−0.8465	0.6179	0.4706

**MoS**_**2**_ **-QD-NH**_**3**_													
S_33_–N_37_	76	0.5881	0.1634	0.3390	−0.6946	−0.2696	0.6946	0.2551	−0.1634	−0.2368	−0.3154	0.2186	0.3317
S_32_–N_37_	53	0.4143	0.1344	0.2593	−0.7679	−0.1825	0.7679	0.1370	−0.5267	−0.4012	−0.1805	0.1565	3.4985
Mo_8_–S_35_⋯H_39_	61	0.9991	0.2417	0.5461	−0.5823	−0.4879	0.5823	0.5585	0.1118	−0.8145	−0.8475	0.4079	0.0404

From the calculated values of *ρ*(*r*), ∇^2^*ρ*(r), *V*(*r*), *G*(*r*), *E*(*r*) and *λ*_2_ for the MoS_2_ doped surface and the adsorbed gas summarized in Table 6, negative values of *H*(*r*) were observed from N_40_–N_37_, Mo_8_–S_11_⋯H_37_ and Si_36_–N_38_, indicating that the interactions at these points were covalent; whereas other bond formations had positive values, indicating strong electrostatic bonding. The density of all electrons of the studied surface was observed to be in the order of 0.993 a.u. for B@MoS_2_-QD-NH_3_. The interaction between the nitrogen-doped surface and the adsorbate was observed to be in the range of 0.132 a.u. to 0.173 a.u. for P@MoS_2_-QD-NH_3_ and the density of electrons was observed to be in the range 0.181 a.u. to 0.993 a.u. Similarly, for Si@MoS_2_-QD-NH_3_ interaction was observed to have electron densities in the range of 0.143 a.u. to 0.803 a.u. The bare surface of MoS_2_ was seen to have 0.999 as its density of states. The highest values of the density of electrons indicate the strongest noncovalent interactions in the studied systems. Different ranges in the density of electrons observed and the different topological parameters could be due to differences in the nature of the doped metals. All other parameters presented in Table 6 further confirmed the noncovalent nature of the studied surfaces, as the values observed are in a good agreement with the previous values observed for noncovalent interactions.^65^ The strongest bond in complexes further suggested the reactivity and the sensing ability of the studied surfaces. It very important to point out that hydrogen bonds were also observed from the interaction of the doped surface with the adsorbate, as presented in Table 6. The results for *λ*_1_, *λ*_2_ and *λ*_3_ obtained from the QTAIM studies were further evaluated with the help of NCI analysis, and strong correlation was observed from this study.

### 3.8 Density of states (DOS) analysis

To further investigate and understand the different characteristic and properties between the gas senor ability of MoS_2_ and its B, N, P, and Si doped surfaces, density of states analysis was carried out in this present work and the result presented in Fig. 6 show the density of states plotted in the ranges of −2.0 a.u. to 25.0 a.u. and −2.0 a.u. to 27.0 a.u. for the interacted adsorbent–adsorbate interaction. This density of states was carried out to analyze the mechanism and sensing ability of the studied systems in order to determine the surface that best detects NH_3_ gas. Not only was the mechanism studied but also the adsorption properties and characteristics of some selected doped surfaces like B@MoS_2_-NH_3_, N@MoS_2_-NH_3_, P@MoS_2_-NH_3_, Si@MoS_2_-NH_3_ and the bare surface of the MoS_2_ monolayer in detecting NH_3_ gas molecules. The DOS plots reveal that the electronic state near the Fermi level increases as the result of the doped atoms, corresponding to the increase in the HOMO–LUMO gap of the studied systems, indicating the strength of the interaction between the surfaces and the adsorbate.^66^ It is important also to point out that due to the large scale of the non-overlapping area, the plots observed in Fig. 6 are similar, due to the morphology of the surfaces. Sulfur atoms in all the interaction between the doped surfaces and the gas molecule prove the strong chemical interaction, and also show the most intense peaks. From the plotted density of states, and the observation made earlier that the DOS near the Fermi level were relatively wide, which implies that the highest occupied levels have many electrons that can seldom transit to the conducting band, and due to the wide Fermi levels observed, the conductivity of the titled molecules was observed to be good and hence the doped atoms are good sensing materials. Multiwfn software was employed for characterization of the DOS of the investigated system.^67^ From the DOS plot, TDOS represents the total density of states, PDOS is the partial density of states, which is contributed by the individual orbitals present in the studied compound, while OPDOS is the overlapping partial density of states curve. The OPDOS observation here shows antibonding characteristics, which could be better explained on the basis of the unfavorable overlap in the orbital phase. It is clear that occupied frontier MOs are solely contributed by the covalently bonded sulfur atoms. The axes on the left-hand side correspond to TDOS and PDOS, while the one on the right-hand side corresponds to OPDOS. The red, blue, pink, and green discrete lines represent the PDOS of molybdenum, sulfur, nitrogen, respectively.

**Fig. 6:** Density of states (DOS) plots for B@MoS_2_-NH_3_, N@MoS_2_-NH_3_, P@MoS_2_-NH_3_Si@MoS_2_-NH_3_ and MoS and MoS_2_–NH_3_ obtained from a multifunctional wave function analyzer.

### 3.9 Transport and electronic properties

Understanding the changes in the electronic properties of an MoS_2_ pure surface and its doped surface upon adsorption of NH_3_ is very crucial, as it help in predicting the sensing applications of these surfaces. To fully compare the electronic properties of MoS_2_ and its doped surface, the geometric energy of the modelled systems was minimized, being brought to a minimum *via* geometric optimization of the systems. The optimized structures are presented in Fig. 1 and 2 and the detailed electronic properties of the modelled systems were calculated at different levels of theory. This is due to the inability of some nitrogen-based molecules with a fully substituted nitrogen atom to partake in the second stage of the reaction. For this we calculated the electronic density of states (DOS), the partial density of states (PDOS), and the total density of states (TDOS) and the figures are presented in Fig. 6. A discrete DOS across the Fermi level for all the modelled systems B@MoS_2_-NH_3_, N@MoS_2_-NH_3_, P@MoS_2_-NH_3_, Si@MoS_2_-NH_3_ and the bare surface of MoS_2_ monolayer in detecting NH_3_ gas molecules was observed, demonstrating their metallic nature.^68^ Furthermore, in the neighborhood of the Fermi level, P@MoS_2_-NH_3_ has the maximum availability of electronic states, although the difference in DOS for all the modelled systems is not significant. As can be seen in Fig. 6, a number of peaks can also be seen in the valence and conduction bands. As a result, the observed NH_3_ aided variations in the electronic properties of the DOS of MoS_2_ and its doped surfaces are significant enough to be used for sensing applications.

#### 3.9.1 Band structure and charge mobility

An MoS_2_ monolayer is observed to possess nonzero band gaps of *E*_g_ = 3.3105, 1.1478, 0.9404 and 2.7241 eV calculated at different levels of theory, ωB97XD, PBE1PBE, B3LYP and M06-2X respectively, consisting of the valence band maximum (VBM) and the conduction band minimum (CBM) at two midpoints along the symmetric lines, according to Fig. 4. The carrier mobility on the other hand is an important parameter that is used in dictating the electronic applications of an MoS_2_ monolayer as a potential senor material for NH_3_ gas.^69^ From a literature review, inorganic semiconductors consist of electron–phonon scattering, which dominates the intrinsic carrier mobility, and acoustic phonon scattering, which dominates carrier mobility. Carrier mobility can be calculated using deformation potential theory.^70^ An analytical expression for the carrier mobility (*t*) for a one-dimensional system was derived by Beleznay *et al.*,^71^ which has been employed in this study to study the charge transport in the MoS_2_ surface and the NH_3_ molecule, calculated using eqn (10).10where (*Φ*) is the charge mobility, *C* is the stretching modulus given as  and *Z*_0_ is the lattice constant. *T* is the temperature, taken in this study to be 298 K. M* is the effective mass of the charge carrier, which is calculated from M* = *η*^2^[d^2^*E*(*K*)/d*k*^2^]^−1^ at the VMB and CMB of the band structure. *E*_1_ is the deformation potential constant due to the quasi-static deformation of the MoS_2_ monolayer, which indicates the shift of the band edge energy. *E*_1_ = d*E*_edge_/d*ε*, where *E*_edge_ stands for the value of the CBM (for electrons) or VMB (for holes).^72^

## 4. Conclusions

Theoretical calculations using the density functional theory (DFT) model were used in this work to study the adsorption mechanism of MoS_2_ and its doped surfaces B@MoS_2_-NH_3_, N@MoS_2_-NH_3_, P@MoS_2_-NH_3_, and Si@MoS_2_-NH_3_ in order to provide adequate information on the sensitivity, selectivity and conductivity of the model sensor material. A monolayer of MoS_2_, purely made from a honeycomb sheet of molybdenum atoms covalently sandwiched between two honeycomb sheets of sulfur atoms and Mo atoms, together with its doped surfaces, was first optimized using high-level theory and the geometric parameters together with the electronic properties of the studied systems were estimated. From the structural properties, P@MoS_2_-NH_3_ had the longest bond length before and after adsorption of NH_3_ molecules and N@MoS_2_-QD-NH_3_ had the shortest bond length (1.419 Å), which could be attributed to the higher electronegativity of the doped atom compared to its counterpart. From the electronic properties, P@MoS_2_-NH_3_ was observed to have a very small gap between the conduction band and the valence band, indicating an increase in conductivity of the systems. The energy gap was observed to decrease when the gd3bj dispersion correction was employed. From natural bond orbital analysis, the delocalization of the π system within the studied surface was also evaluated using occupancy of the Lewis donor and the acceptor in which P@MoS_2_-NH_3_ was observed to have the highest occupancy that corresponded to its lowest energy gap. Comparative adsorption energy was evaluated from which the most negative values were obtained from ωB97XD compared to the other functionals. P@MoS_2_-NH_3_ was observed to have the highest negative adsorption energy compared to the other doped surfaces. From adsorption mechanistic studies, we observed that after doping, the dipole moment was observed to increase significantly based on the charge separation in the doped atoms. Noncovalent interaction within the studied surface was confirmed by QTAIM and NCI. From this study P@MoS_2_-QD-NH_3_ was observed to have stronger noncovalent interaction compared to other doped surfaces, which was further confirmed by the higher density of electrons and the Laplacian of electron density. These results show that a P@MoS_2_-QD-NH_3_ doped surface is more conductive than the other doped surfaces.

## Author contributions

Hitler Louis: project conceptualization, design, and supervision. Terkumbur E. Gber: writing, results extraction, analysis, and manuscript first draft. Benjamin Etinwa and Benjamin Innocent: manuscript revision, review, and proofreading. Fredrick C. Asogwa and Ededet A. Eno: manuscript proofreading and Aniekan E. Owen and Adedabo Adeyinka: resources, review, and editing.

## Conflicts of interest

All authors declare zero financial or inter-personal conflict of interest that could have influenced the research work or results reported in this research paper.

## Supplementary Material

RA-012-D2RA04028J-s001
